# Neutrophils: As a Key Bridge between Inflammation and Thrombosis

**DOI:** 10.1155/2022/1151910

**Published:** 2022-11-09

**Authors:** Pengxiang Xu, Liuyan Xin, Xiaoping Xiao, Yong Huang, Chuanming Lin, Xiaofang Liu, Haiyan Wei, Rong Xu, Yijian Chen

**Affiliations:** ^1^The First Affiliated Hospital of Gannan Medical University, Ganzhou 341000, Jiangxi, China; ^2^Ganzhou Key Laboratory for Drug Screening and Discovery, School of Geography and Environmental Engineering, Gannan Normal University, Ganzhou 341000, Jiangxi, China

## Abstract

Immunothrombosis is a mechanism of defense of the organism against pathogenic microorganisms that increases their recognition, limitation, and clearance and is part of the innate immune defense. Physiological immunothrombosis is beneficial to the body against the invasion of pathogenic microorganisms, but when immunothrombosis is out of control, it is easy to cause thrombotic diseases, thus, causing unpredictable consequences to the body. Neutrophils play a pivotal role in this process. Understanding the mechanism of neutrophils in immune thrombosis and out-of-control is particularly important for the treatment of related thrombotic diseases. In this review, we studied the role of neutrophils in immune thrombosis and each link out of control (including endothelial cell dysfunction; activation of platelets; activation of coagulation factor; inhibition of the anticoagulation system; and inhibition of the fibrinolysis system).

## 1. Introduction

Neutrophils are phagocytes derived mainly from bone marrow and extramedullary myeloid progenitors, which mainly play a role in resisting the invasion of pathogenic microorganisms in normal bodies and belong to the innate immunity of the body [1]. Recent research has shown that neutrophils are also implicated in thrombosis in the body. When pathogens invade the body, they can be directly recognized, phagocytized, and removed by neutrophils in order to obtain the immune defense effect. However, when the invading pathogen exceeds the phagocytic capacity of local neutrophils, too many pathogens will induce neutrophil cell death (NETosis), a form of death distinct from necrosis and apoptosis [2], during this process, the activities of neutrophil elastase (NE), myeloperoxidase (MPO), and nicotinamide adenine dinucleotide phosphate oxidase (NADPH) increased, It eventually leads to degradation of histone, DNA decondensation, nuclear rupture, membrane lysis, and the release of intracellular chromatin filaments into extracellular neutrophils to form a neutrophil extracellular trap (NET) [3, 4]. The formation of NET can make the body more resistant to pathogenic microorganisms that invade the body, thus enhancing the immune function of neutrophils in the body, but at the same time, the formation of NET can also activate platelets and coagulation factors and promote the formation of thrombus in the body [5]. Immunothrombosis is named for the first time by Engelmann and Massberg It is a physiological thrombus mediated by immune cells and thrombus-related molecules to resist the invasion of pathogenic microorganisms. It can not only limit the pathogenic microorganisms that invade the body but also prevent them from spreading further through blood vessels. But can also enhance the function of the immune system to recognize and eliminate pathogenic microorganisms [6]. While proper immunothrombosis are beneficial to the body, abnormal or excessive activation of immunothrombosis can lead to serious cardiovascular diseases such as myocardial infarction, stroke, venous embolism, and ischemic damage to other vital organs, often causing fatal damage to the body [7].

## 2. Endothelial Cells and Neutrophils

Endothelial cells (ECs) belong to monolayer flat epithelial cells, which mainly regulate plasma-tissue material exchange, participate in blood coagulation, regulate vascular tension and recruit related blood cells [8]. In addition, some studies have shown that ECs belongs to untraditional immune cells, which can be activated by pathogenic microorganisms invading the body through pattern recognition receptors, and then secrete related cytokines (G-CSF, IL-8, TNF-*α*, and so on), chemokine (CXCL1, ACKR1, and so on), adhesion molecules (CD62E/P, VCAM-1, PECAM, ICAM-2, and so on) to activate and recruit neutrophils in circulation [9]. Sepsis caused by the invasion of pathogenic microorganisms can damage the glycocalyx layer of endothelial cells through glycosaminoglycan (GAG) degradation and core membrane binding proteoglycan (PG) cleavage, while the injury of the endothelial cell glycocalyx layer will enhance the adhesion and interaction between endothelial cells and neutrophils, and the degraded glycocalyx fragments can also enhance the inflammatory response in vivo, thus, activating a large number of neutrophils [10]. Activated neutrophils reach the site of inflammation or infection through the recruitment of chemokines, release a large number of cytokines, phagocytize pathogens with the help of complement, and then, kill and decompose pathogens in intracellular phage particles so as to play the role of innate immunity [5]. When the invading pathogen exceeds the phagocytic capacity of a limited number of local neutrophils, in order to prevent the body from further invasion by pathogens, neutrophils lysis releases NET rich in nuclear components (histones, DNA) and granules (elastase, myeloperoxidase, cathepsin, and so on). The network structure formed by NET limits the pathogen to the site of inflammation or infection [11], which plays an important role in the process of innate immunity. NET can act as the body's defense structure, but it can also have harmful effects on surrounding tissues. Activated neutrophils can release a large number of relevant complement factors such as P, B, and C3. When NET is formed, these complement related components can be deposited on the reticular structure of NET, and the activated complement, finally, forms a membrane attacking complex to damage the corresponding endothelial cells [12]. Moreover, the formation of NET can also promote the activation of endothelial cells and lead to their dysfunction. Histones and matrix metalloproteinases (MMPs) released during the formation of the reticular network have been found to be highly toxic to endothelial cells [13–15]. In addition, some pathogens limited by NET (such as pathogen *V. harveyi*, *P. fluorescens,* and *E. tarda*) are not completely killed and can still replicate slowly and continuously stimulate inflammation and complement activation [16]. Proinflammatory factors such as activated complement C3a, C5a, and mannose-binding lectin (MBL) can recruit more inflammatory cells such as neutrophils for infiltration [17], exacerbating the local inflammatory response and sustaining damage to endothelial cells. It has also been shown that complement C3 plays an important role in the process of platelet activation and deposition of fibrin [18]. Furthermore, activated neutrophils produce large amounts of reactive oxygen species (ROS) through a multiprotein membrane-bound NADPH oxidase complex, which are released to the site of inflammation during NET formation and induce the production of more NET while killing bacteria and promoting the production of proinflammatory factors as well as damaging the glycocalyx layer of endothelial cells [19–21]. The lysis of neutrophils during NET formation releases large amounts of ROS-containing mitochondria, histones, microsomes, and DNA, which can further promote inflammation and damage endothelial cells. Following damage to the endothelium, the functional barrier of the endothelium is disrupted and the corresponding increase in adhesion molecules and chemokines enhances neutrophil adhesion, exposing the tissue factor (TF), and von Willebrand factor (vWF) originally covered by the barrier, which in turn activates coagulation and ultimately interacts with the NET to cause immune thrombosis.

## 3. Platelets and Neutrophils

Platelets are key molecules in the process of physiological hemostasis and pathological thrombosis in the body and are fragments of nucleated cells produced by the lysis of bone marrow megakaryocytes. Recent studies have shown that platelets also play an important role in the immune system (identifying and limiting pathogens, enhancing neutrophil activation and participating in immunothrombosis, and so on.). Under normal physiological conditions, platelets in the blood exist independently of neutrophils, and when a pathogen invades the body, it first causes local inflammation by pattern-recognizing receptor activation and destruction of endothelial cells. The formation of inflammation will lead to the deposition of fibrinogen in the plasma, and some circulating platelets are activated by the deposited fibrinogen and form platelet pseudopods that continuously scan and promptly detect sites of bacterial infection within the vascular endothelium, subsequently recruiting more platelets to activate and rapidly recruit and migrate via integrin receptors to accumulate on the endothelial cell surface at that site, trapping the pathogen and preventing its further spread [22]. Activated platelets release a large number of chemokines and adhesion molecules to recruit circulating neutrophils. Activated platelets produce dioxolane A3-phosphatidylethanolamine (DXA3-PE), 5-hydroxytryptamine (5-HT), and other substances to stimulate the expression of integrins on the surface of neutrophil membranes and improve neutrophil adhesion [23, 24], making it easier for neutrophils to adhere to activated platelets and endothelial cells. In addition to increasing the expression of the integrin subtype CD11b molecule on the surface of neutrophils, platelet-derived 5-HT promotes degranulation of neutrophils, leading to increased release of myeloperoxidase (MPO), hydrogen peroxide (H2O2), tumor necrosis factor alpha (TNF-*α*) and other substances, ultimately leading to an increased inflammatory response [24]. In addition, the platelet 5-HT metabolite 5-hydroxyindoleacetic acid (5-HIAA) can also promote the expression of neutrophil GPR35, and thus, the recruitment of neutrophils to sites of inflammation [25]. In addition, studies have shown that dengue virus can activate platelets through clec2, and activated platelets release extracellular vesicles (EVs) and form a DV-EVs complex with DV to further activate clec5a and TLR2 in neutrophils and macrophages, thus, inducing the formation of NET and the release of a large number of inflammatory factors [26]. Maugeri et al. have shown that platelet-derived particle-associated high mobility group protein b1 (HMGB1) can interact with neutrophils to promote neutrophil activation and autophagy to produce NET [27–30]. Platelets recruit and activate neutrophils through the above methods. In addition, neutrophils can also be directly activated by pathogens through pattern recognition receptors. After neutrophils are activated, they will produce a large number of inflammatory factors, in which IL-6 can act on the liver, stimulate the liver to produce more thrombopoietin (TPO), and make the body produce more platelets and release them into the blood circulation [31]. Moreover, integrin *α*9*β*1 was also found to be highly expressed on activated neutrophils and to play an important role in mediating platelet aggregation, in which the authors prepared myeloid-specific integrin *α*9−/− mice and found a significant reduction in neutrophil-mediated platelet aggregation in these mice [32]. In contrast, NET produced by neutrophil lysis can promote the deposition of fibronectin and vWF and provide a scaffold for adhesion of activated platelets [33, 34], And the histones released during NET formation can bind directly to platelets and induce platelet calcium inward flow and also recruit adhesion proteins such as fibrinogen to induce platelet aggregation [35]. In addition, neutrophils can bind directly to activate platelets. When platelets are activated, they release P-selectin stored in *α* granules and increase the expression of P-selectin on its membrane surface. Through P-selectin binding glycoprotein ligand (PSGL), neutrophils directly bind to neutrophils and activate neutrophils to form neutrophils-platelet complexes (platelet-neutrophil-complexes, PNC) [36]. On the other hand, the platelet membrane can form flow-induced PRotrusions (FLIPRs) under high cytoplasmic calcium and shear forces of blood flow P-selectin exposed to the surface of processes can bind to PSGL on the surface of the neutrophil membrane, further promoting the recruitment and activation of neutrophils and promoting the formation of PNC [37]. The formation of PNC not only recruits and activates neutrophils and promotes their lysis to release NET, but also promotes the release of ROS from neutrophils and damages surrounding endothelial cells and other immune cells, further aggravating inflammation and thrombosis [38–40]. In conclusion, the interaction between neutrophils and platelets jointly promotes the formation of immunothrombosis. When immunothrombosis is out of control, it will aggravate the immunothrombosis formation process and eventually lead to a continuous increase in body injury.

## 4. Coagulation Factors and Neutrophils

Similar to platelets, coagulation factors also play a role in hemostasis and thrombosis in the body, forming an exogenous coagulation pathway with TF as the trigger and an endogenous coagulation pathway with factor XII (FXII) as the trigger, through which the coagulation cascade in the body is triggered, leading to the formation of fibrin and cross-linking with platelets to promote hemostasis or thrombosis. Recent studies have shown that coagulation factors also have immune-related functions and can interact with neutrophils to promote immune thrombosis. FXII as a trigger condition for the endogenous coagulation pathway was found to promote neutrophil recruitment and migration and NET release by upregulating the expression of integrin *α*M*β*2 on the surface of neutrophils and increasing their intracellular calcium ion concentration and extracellular DNA release, as verified by Stavrou EX et al. Using an FXII −/− knockout-deficient mouse model [41]. FXII or thrombin activated factor XI (FXI) has been found to increase the phagocytosis of neutrophils in mouse models of *Streptococcus pneumoniae* or *Klebsiella pneumoniae pneumonia*, thus, increasing the immune function of neutrophils [42]. In a study of patients with COVID-19, TF expression was found to be significantly elevated on the patient's neutrophils, in addition to the release of NET carrying active TF by neutrophils, and the complement C3 inhibitor comptincp40 was found to reduce neutrophil TF expression, suggesting that high neutrophil TF expression in this patient was associated with complement C3 [43]. In addition, a recent study has shown that fibronectin deposited in the oral mucosa can promote neutrophil activation via the integrin receptor *α*M*β*2 and promote the production of reactive oxygen species by neutrophils and the release of NET [44]. It is clear that some coagulation factors can increase the activation of neutrophils. On the other hand, neutrophils can release *α*-defensins (*α*-defs) when they are activated. Under pathological conditions, the substance can directly bind to fibrin, promote the polymerization of fibrin, increase the quality of fibrin, and hinder the dissolution of fibrin [45]. In a study of patients with systemic lupus erythematosus, it was found that neutrophils in lupus erythematosus patients showed a higher level of autophagy than normal people, and were more likely to lysis and release NET rich in TF and IL-17A [46]. In addition, it was found that the treatment of human endothelial cells with purified NET could increase the expression of TF mRNA and the activity of TF in endothelial cells [14], In addition, it has been shown that the inflammatory factor TNF-*α* can also promote TF expression in endothelial cells, and the authors found that 15-epi-lipoxin A4 can inhibit this process [47]. It is well known that FXII can be activated by negatively charged surfaces to initiate the coagulation cascade via the endogenous coagulation pathway, and that in addition to the formation of negatively charged NET, a large amount of negatively charged material such as mitochondrial DNA is also released during NET formation [48], and that these negatively charged surfaces will activate FXII. Apart from that, NETs as extracellular DNA can promote the deposition of fibrinogen on NETs, thereby increasing the protein formation of fibrils [49]. Coagulation factors promote the activation of neutrophils through many of the pathways mentioned above. Activated neutrophils, as well as NET released by neutrophil lysis, in turn activate endogenous and exogenous coagulation pathways, leading to fibrin formation. Fibrin, in turn, cross-links with neutrophils and platelets to promote the formation of immunothrombosis.

## 5. Anticoagulation, Fibrinolytic System, and Neutrophils

In addition to the participation of the cells and molecules mentioned above, the dysfunction of the anticoagulation system and the fibrinolysis system is also involved in the process of immunothrombosis. As mentioned above, when a large number of pathogens invade the body through the vascular system, a large number of neutrophils are recognized and recruited by endothelial cells, resulting in inflammation, and eventually a large number of endothelial cells are damaged. The integrity of endothelial cells is an important part of the anticoagulant system. It can express a large number of natural anticoagulants such as glycosaminoglycan, endothelial protein C receptor, tissue factor pathway inhibitors and thrombomodulin and secrete anticoagulant molecules such as tissue plasminogen activator (*t*-PA), urokinase plasminogen activator (u-PA), and nucleoside diphosphate hydrolase-1 (CD39) [50, 51]. Massive damage to endothelial cells eventually leads to a decrease in the production of these anticoagulant substances. When the endothelial cell protein C receptor is damaged, its ability to bind to protein C will also decrease, eventually promoting blood coagulation and inflammation [52]. In addition, some studies have found that the expression of thrombomodulin and protein C receptor on endothelial cells in COVID-19 patients is significantly decreased, and its mechanism is related to the infiltration of immune cells in the lungs of COVID-19 patients [53]. However, some people have found that heparin, as a natural anticoagulant, can bind to platelet activating factor 4 (PF4) and modify it to form an immune complex (heparin-induced thrombocytopenia immune complex, HITIC) by IgG. The immune complex can directly activate platelets and neutrophils through Fc*γ* receptor subtype Fc*γ*RIIa on the cell membrane, promote platelet release of particles and related procoagulant factors, stimulate neutrophils to form NET, and enhance their interaction [54, 55]. In addition, the immune complex activates complement via the classical pathway and promotes complement deposition on the surface of neutrophils, and the activation of complement further increases the interaction of the immune complex with neutrophils and platelets [56]. One study found a significantly higher incidence of HIT IC in patients with COVID-19 [57], suggesting that increased immune responses and excessive platelet activation increase this process in heparin. The presence of plasminogen activator inhibitor type-1 (PAI-1) inhibits the production of fibrin, a process that is essential for the maintenance of coagulation homeostasis, and it has recently been shown that PAI-1, in addition to inhibiting fibrin production, also induces neutrophil activation recruitment [58], it can induce changes in the conformation of *β*2 integrins on the surface of neutrophils and increase their affinity, ultimately increasing neutrophil recruitment and infiltration at the site of damage [59]. Tissue factor pathway inhibitor 2 (TFPI-2) inhibits the exogenous coagulation pathway activated by tissue factor, while elastase released during NET production by neutrophil lysis can degrade TFPI-2 by cleaving it and thus rendering it less anticoagulant [60]. In addition, NE can also inactivate plasminogen to reduce plasminogen production and form a NE-DNA complex with DNA released from neutrophils during NET formation. The complex can reduce the concentration of local plasminogen and reduce plasminogen production, resulting in reduced fibrin degradation [61]. During NET formation, histones are also released into the plasma in large quantities, which cross-link with fibrin and induce changes in fibrin conformation, accelerating the aggregation of fibrinogenic fibrils and causing them to form thicker fibrin to prevent their lysis by fibrinolytic enzymes [62]. It has also been shown that heparin and DNA, as anionic substances, can also inhibit fibrinolysis and increase the mechanical stability of fibrin [63, 64]. Ultimately, activated neutrophils compromise the body's anticoagulant and fibrinolytic systems through this series of pathways, ultimately leading to the formation of immunothrombosis.

## 6. Conclusions

The formation of immunothrombosis belongs to the normal physiological phenomenon of the body against harmful stimuli (such as pathogens), which can limit the further spread of pathogens, which is undoubtedly beneficial to the body. After exerting immune function, a small amount of NET in immunothrombosis can be cleared by macrophages and DNA enzyme [65, 66], and under the action of related fibrinolytic enzymes, pathogens, and immunothrombosis can be cleared in time to restore the homeostasis of the body. However, when a large number of pathogens invade the body, the resulting immunothrombosis is not cleared in time and interacts with endothelial cells, platelets, coagulation factors, anticoagulants, and fibrinolytic substances through the above pathways to form a harmful cycle that is constantly amplified and eventually leads to uncontrolled immunothrombosis (Figure 1). NET released by neutrophil lysis also plays a crucial role in this process, and exogenous DNA enzyme have been shown to reduce NET already formed in plasma [67]. It is suggested that exogenous DNA enzyme therapy has the potential to immune thrombosis out of control. However, Quan et al. have shown that DNA enzyme treatment can affect the survival rate of tumor-bearing mice. The authors suggest that this is due to increased susceptibility to sepsis in mice [68]. Therefore, the questions of whether NET degradation leads to bacterial proliferation and when is the most appropriate time to use the DNA enzyme need to be further addressed, and the specific signal transduction mechanisms involved in NET formation are still under-researched and need to be further investigated. Finally, how to break these cellular and molecular interactions that together activate this harmful cycle and reduce the formation and increase the degradation of NET during this process will also be a key aspect of future treatments for this type of thrombotic disease.

## Figures and Tables

**Figure 1:** When pathogens invade the body, a small number of pathogens will be cleared by neutrophils and the body will return to normal. However, when the pathogen invading the body exceeds the clearance capacity of neutrophils, the formation of neutrophil lysis and the release of NET occur. NET activates platelets, endothelial cells, coagulation factors, and damages the body's anticoagulation and fibrinolysis systems, making the body in a hypercoagulable state. Activated neutrophils can also interact with activated platelets, endothelial cells, coagulation factors, anticoagulant, and fibrinolytic factors to further accelerate thrombosis and eventually lead to immune thrombosis.

## Data Availability

The data that support the findings of this study are available from the corresponding author upon reasonable request.
